The article "Facial Emotion Recognition Using a Novel Fusion of Convolutional Neural Network and Local Binary Pattern in Crime Investigation" was retracted in 2026. Reasons: suspected computer-generated content; concerns about the data; concerns about the peer review; concerns about the citations.

# Facial Emotion Recognition Using a Novel Fusion of Convolutional Neural Network and Local Binary Pattern in Crime Investigation

**DOI:** 10.1155/2022/2249417

**Published:** 2022-09-22

**Authors:** Dimin Zhu, Yuxi Fu, Xinjie Zhao, Xin Wang, Hanxi Yi

**Affiliations:** ^1^School of Law, Zhejiang Gongshang University, Hangzhou, Zhejiang Province 310000, China; ^2^Department of Science and Technology, Beijing Normal University-Hong Kong Baptist University United International College, Zhuhai 519087, China; ^3^School of Software and Microelectronics, Peking University, Beijing, China; ^4^Behavioural Science Institute, Radboud University, Nijmegen 6525 GD, Netherlands; ^5^Division of Biopharmaceutics and Pharmacokinetics, Xiangya School of Pharmaceutical Sciences, Central South University, Changsha 410000, China

## Abstract

The exploration of facial emotion recognition aims to analyze psychological characteristics of juveniles involved in crimes and promote the application of deep learning to psychological feature extraction. First, the relationship between facial emotion recognition and psychological characteristics is discussed. On this basis, a facial emotion recognition model is constructed by increasing the layers of the convolutional neural network (CNN) and integrating CNN with several neural networks such as VGGNet, AlexNet, and LeNet-5. Second, based on the feature fusion, an optimized Central Local Binary Pattern (CLBP) algorithm is introduced into the CNN to construct a CNN-CLBP algorithm for facial emotion recognition. Finally, the validity analysis is conducted on the algorithm after the preprocessing of face images and the optimization of relevant parameters. Compared with other methods, the CNN-CLBP algorithm has higher accuracy in facial expression recognition, with an average recognition rate of 88.16%. Besides, the recognition accuracy of this algorithm is improved by image preprocessing and parameter optimization, and there is no poor-fitting. Moreover, the CNN-CLBP algorithm can recognize 97% of the happy expressions and surprised expressions, but the misidentification rate of sad expressions is 22.54%. The research result provides data reference and direction for analyzing psychological characteristics of juveniles involved in crimes.

## 1. Introduction

The popularization of the Internet has caused immense changes in the social environment, resulting in a significant impact on the outlook on life and values of young people, followed by psychological problems that cannot be ignored [1, 2]. Therefore, it is of vital significance to seek a method that can accurately judge the psychological state and psychological characteristics of minors. In the context of the burgeoning artificial intelligence technology, the development of deep learning and natural language processing technology provides technical support for the solution to this problem [3–5]. In the field of psychological analysis, emotion recognition is also called emotion analysis, which is used to analyze complex emotional states [6]. Facial expression is an external and intuitive reflection of emotion, and facial expression recognition technology can identify human emotional state. So far, many research results have been achieved on the application of deep learning to facial emotion recognition of excellent applicability.

The article "Facial Emotion Recognition Using a Novel Fusion of Convolutional Neural Network and Local Binary Pattern in Crime Investigation" was retracted in 2026. Reasons: suspected computer-generated content; concerns about the data; concerns about the peer review; concerns about the citations.

The conventional methods of facial emotion recognition usually collaborate with feature extraction, feature classification, and data dimension reduction algorithms and put forward stringent requirements for the running state of algorithms at each stage [7]. Neural network models are constantly improving and developing with the improvement in computers. On the one hand, artificial intelligence technology is primarily employed for the perception of emotion. Besides, the progress of neural network models and other technologies also provides a new direction and idea for solving problems in common facial emotion recognition. On the other hand, facial emotion recognition technology has mainly experienced three stages of development. In the primary stage, the identification of facial expressions is realized through the facial action coding system. In the second stage, facial emotion recognition is manifested in systematic recognition, including three steps, namely, information collection, feature extraction, and expression recognition. The methods used in this stage primarily contain support vector machine (SVM), Gabor wavelet, and Local Binary Pattern (LBP). However, in this stage, the recognition accuracy needs to be enhanced because the facial emotion recognition excessively depends on feature algorithm classifiers and explicit expression features. In the last stage, the deep learning algorithm is the most dominant approach to facial emotion recognition. Its most predominant feature is that it can input and output relevant data through the deep learning model instead of artificial classifiers, and this method significantly alleviates local optimization. Among diversified deep learning algorithms, the convolutional neural network (CNN) algorithm can achieve excellent performance in image recognition and attains higher recognition accuracy than the conventional algorithms.

However, the current CNN model is incompetent. Therefore, the CNN model is optimized before recognizing facial expressions and analyzing facial emotions. Specifically, a facial expression recognition algorithm is proposed by integrating the CNN model and Central Local Binary Pattern (CLBP) to analyze and identify facial expressions. It is expected to provide reference for the optimization of deep learning algorithm for facial expression recognition and preliminarily explore the correlation between facial expression recognition and psychological feature analysis.

The article "Facial Emotion Recognition Using a Novel Fusion of Convolutional Neural Network and Local Binary Pattern in Crime Investigation" was retracted in 2026. Reasons: suspected computer-generated content; concerns about the data; concerns about the peer review; concerns about the citations.

The main contributions of this paper are summarized as follows:

1. A fusion CNN model is constructed for facial emotion recognition. The comparative analysis indicates that the overall performance of the model reported here is better than the traditional LBP model, LeNet-5 model, and VGGNet model. The highest recognition accuracy of happy expressions of the fusion CNN model attains 98.61%, which is better than 94.11% of the VGGNet model.
2. A hybrid CNN-CLBP facial emotion recognition algorithm is proposed based on optimized CLBP algorithm. This algorithm has outstanding performance in facial expression recognition, and the average recognition rate of happy expressions and surprised expressions is 97%.
3. The research results provide a feasible direction for the analysis of psychological characteristics based on emotion recognition.

## 2. Literature Review

Some scholars have made efforts into the recognition of facial expressions. For instance, Fan and Tjahjadi proposed a facial expression recognition framework by combining CNN and handcrafted features. They found that the neural network could achieve brilliant recognition effects by extracting texture information from facial patches, and the introduction of CNN had a promoting effect on facial expression recognition [8]. Reddy et al. put forward an organic combination of deep learning features and the manual facial expression recognition method. They verified the applicability of this method in the wild scenes in experiments, which revealed the effectiveness of the recognition method under the combination of deep learning and manual production [9]. Liang et al. emphasized that the traditional handcrafted facial representations could only reveal shallow features. To break out this limitation, they proposed a new facial expression recognition method based on patches of interest, the Patch Attention Layer of embedding handcrafted features, to learn the local shallow features of each patch on face images. They finally proved the effectiveness of the method in their study [10]. Jain et al. (2018) built a hybrid convolutional-recursive neural network for facial expression recognition, which extracted information on face images through the combination of convolutional layer and Recurrent Neural Network (RNN) in view of the time correlations in images [11]. Avots et al. identified human emotions through analyzing audiovisual information. Besides, they classified the emotions on face images using different datasets as test sets, Viola-Jones face recognition algorithm, and CNN (AlexNet) [12]. Li et al. constructed a two-dimensional principal component analysis network via deep learning based on L1 norm for face recognition, tested it on some facial image database, and found that the network was robust [13]. Bernhard et al. stated that emotions had a significant influence on decision-making of humans, and hence, they applied deep learning to improve emotion recognition results. They found that the performance of RNNs and transfer learning was better than traditional machine learning, which had great inspirations on emotion computing application [14]. Kumar et al. discussed the modeling of abnormal facial expressions based on computer vision tasks and emotional deviations. They found that deep CNN could play an essential role in the training and classification of facial expressions, which provided a new visual modeling method for visual surveillance systems [15]. Mishra et al. employed CNN to recognize different emotions and intensity levels of human faces, which provided the basis and support for future research on computer emotion recognition [16].

The article "Facial Emotion Recognition Using a Novel Fusion of Convolutional Neural Network and Local Binary Pattern in Crime Investigation" was retracted in 2026. Reasons: suspected computer-generated content; concerns about the data; concerns about the peer review; concerns about the citations.

In summary, the traditional manual methods are no longer suitable for the current research on facial expression recognition, but deep learning can significantly improve the recognition effectiveness of facial expression, especially the hybrid model. Although some achievements have been made in the previous studies of facial expression recognition, there are few studies combining it with psychological analysis.

## 3. Materials and Methods

### 3.1. CNN Model Based on Deep Learning

CNN is a typical neural network based on deep learning, which can reduce the resolution of features, thereby showing significant advantages in the extraction of image features and analyzing modal image data [17, 18]. CNNs are primarily composed of the convolution layer, the pooling layer, and the fully connected layer [19]. Among them, the convolution layer is the most significant component distinguishing the CNN from other neural networks, which can perform convolution operations on image features to obtain various forms of feature maps and all the edge information on the image simultaneously. Besides, the convolution layer of CNNs is mainly characterized by functions including local connections, receptive fields, and shared weights, ensuring the high efficiency of CNNs in feature extraction and feature calculation. Meanwhile, it enables the CNN to differentiate different images during feature extraction, thereby optimizing the global extraction effect and reducing the training parameters of CNN through shared weights [20]. This layer highlights the initial information about the image and significantly lessens the calculative burden of the model. Consequently, the matching rate of the entire training process is greatly improved [21]. The fully connected layer of the CNN can accomplish the connection to the local features of the image [22], which can be expressed as

(1) $$\begin{array}{c} l_{W,b}\left(x\right)=f\left(W^{T}x+b\right)\text{,} \end{array}$$

where *f* represents the nonlinear activation function, *x* denotes the input, *l* refers to the output, W^T^ signifies the connection weight, and *b* represents the offset.

The article "Facial Emotion Recognition Using a Novel Fusion of Convolutional Neural Network and Local Binary Pattern in Crime Investigation" was retracted in 2026. Reasons: suspected computer-generated content; concerns about the data; concerns about the peer review; concerns about the citations.

The crucial procedure of facial emotion recognition technology based on psychoanalysis is the extraction and classification of image features corresponding to facial expressions. The hidden layer of the CNN completes the extraction of image features and classifies image features by means of classifiers. Among them, Softmax is a widely used classifier, which mainly completes the classification by calculating its probability, as shown in

(2) $$\begin{array}{c} f\left(o_{j}\right)=\frac{e^{o_{j}}}{\sum_{n=1}^{n}e^{o_{k}}}\text{.} \end{array}$$

In equation (2), *n* denotes the number of outputs, and *o*_*j*_ stands for the probability of the output results.

Furthermore, in the neural network model, Dropout can realize the zero processing of some weights.

In short, the CNN is selected for feature extraction and facial emotion recognition based on psychological feature analysis here since it is superior to other neural networks.

### 3.2. Construction of the Facial Emotion Recognition Model Based on Hybrid CNN Network

CNN shows outstanding performance in image feature extraction, but it has some shortcomings. In concrete application scenarios, it is essential to design the CNN structure according to specific recognition tasks. Besides, the model's training is greatly affected by the number of network layers [23–25]. Specifically, the training effect is better with more network layers. As the corresponding weight parameters increase, the entire training duration enlarges. Otherwise, the training process will be shorter. For the recognition task, the deep network's recognition accuracy is better than that of the external network, while the recognition efficiency of the external network is better than that of the deep network. Hence, it is necessary to fully consider the network's recognition accuracy and efficiency for the optimal recognition effect of the neural network. Furthermore, more attention is paid to the recognition accuracy of the proposed model, which is a critical evaluation indicator.  Figure 1 illustrates the structure of CNN with sentences as input.

The article "Facial Emotion Recognition Using a Novel Fusion of Convolutional Neural Network and Local Binary Pattern in Crime Investigation" was retracted in 2026. Reasons: suspected computer-generated content; concerns about the data; concerns about the peer review; concerns about the citations.

VGGNet, AlexNet, and LeNet-5 are common CNN models. The VGGNet model uses convolution kernels of size 3∗3, so it has fewer network parameters and a stronger learning capability than other models with convolution kernels of size 5∗5. However, it has more complex structural components and is not applicable to the classification of small-scale data information [26]. The AlexNet model utilizes multiple graphics processing units (GPUs) to complete the model training, which improves the overall training speed, recognition accuracy, and recognition rate of the model. It plays an essential role in solving the gradient disappearance problem [27, 28]. The LeNet-5 model is the simplest CNN model, which is suitable for low-resolution image recognition and processing of available classification data [29].

### 3.3. Fused CNN Model

#### 3.3.1. VGGNet Model

VGGNet further explains the correlation between the depth and performance of CNN. One of the most prominent contributions of VGGNet model is to reveal that the increase in layers of the CNN model can significantly reduce the error rate and achieve excellent expansion performance and generalization performance, enabling CNN to efficiently extract features from images. The VGGNet model can be regarded as a deeper version of AlexNet model, which is composed of five convolution layers, three full connection layers, and a Softmax output layer. In summary, the model has a relatively simple structure and has a small convolution kernel and pooling kernel, as well as more convolution sublayers and channels. Meanwhile, the model has deeper layers and wider feature maps.

#### 3.3.2. AlexNet Model

The AlexNet model is also a key link to the development of CNN, which realizes the excellent performance of CNN in the field of image classification. The innovation of AlexNet model lies in the smooth application of ReLU activation function and Dropout mechanism, the use of overlapping maximum pooling, the proposal of local response normalization, and the accelerated training of GPU. Among them, the use of ReLU can effectively avoid the occurrence of overfitting and alleviate the interdependence between different parameters to some extent.

#### 3.3.3. LeNet-5 Model

LeNet-5 is a classical CNN model, and its unique structure of convolution-pooling alternation can effectively extract the translation invariant features of the input image. As the name suggests, the LeNet-5 model has five layers in its structure, namely, two convolution-pooling layers and three fully connected layers.

The article "Facial Emotion Recognition Using a Novel Fusion of Convolutional Neural Network and Local Binary Pattern in Crime Investigation" was retracted in 2026. Reasons: suspected computer-generated content; concerns about the data; concerns about the peer review; concerns about the citations.

To sum up, these three models have distinctive excellent performance. Based on this, the advantages of each model are organically integrated to construct a fused CNN model.

### 3.4. Parameter Setting of the Hybrid Neural Network

The facial expression generally accounts for a small proportion of an image, so it is difficult to achieve the optimal effect by applying the above neural network model separately when processing images of such characteristics. As a result, the above three neural network models are combined to construct a fused CNN model for facial emotion recognition, comprising four convolution layers, two pooling layers, two fully connected layers, and a Softmax classification layer.  Table 1 reveals the specific parameter settings of the model. At the initial stage of facial emotion recognition by the hybrid CNN model, the input of the grayscale feature image of facial expressions is completed in the input layer. Next, it is followed by the convolution layer, which corresponds to 1–3 in the following table. Here, the image feature extraction is completed through calculating the output of the region neuron corresponding to the input. Moreover, its back corresponds to the pooling layer 1, which is primarily responsible for the pooling processing on the point corresponding to the maximum value in the region, which is as the values after pooling process. The subsequent layers following pooling layer 1 are convolution layer 4, pooling layer 2, and finally, two fully connected layers and an output layer. Among them, the fully connected layer 1 contains 120 fully connected neurons, and the fully connected layer 2 contains 64 fully connected neurons. The output layer corresponds to the Softmax layer containing six neurons, mainly used to predict the six types of output of human facial emotions.

### 3.5. Facial Emotion Recognition Algorithm Based on Feature Fusion

LBP is an algorithm describing image texture features, and the operator of LBP uses each pixel in the image to calculate the binary mode. In this process, each component pixel in the image is the central pixel, and the corresponding threshold processing is completed through the eight pixels in the neighborhood. When the adjacent pixel is smaller than the central pixel, the adjacent pixel value is 0. Otherwise, the adjacent pixel value is 1 [30, 31]. The operator for image extraction can be expressed as

(3) $$\begin{array}{c} LBP\left(x_{p},y_{p}\right)=\overset{p-1}{\underset{p=0}{\sum }}2^{p}S\left(I_{p}-I_{c}\right)\text{,} \end{array}$$

where (*x*_*p*_, *y*_*p*_) is the information corresponding to the center position in the neighborhood, and *I*_*p*_ represents the pixel value of the image. Meanwhile, *I*_*c*_ signifies the pixel value of other images in the region, and *S* denotes a symbolic function.

The article "Facial Emotion Recognition Using a Novel Fusion of Convolutional Neural Network and Local Binary Pattern in Crime Investigation" was retracted in 2026. Reasons: suspected computer-generated content; concerns about the data; concerns about the peer review; concerns about the citations.

However, the conventional LBP operator only covers a small area within a fixed range. Therefore, the LBP operator has limitations on scenarios of high requirements for textures of different sizes or frequency. It is unsuitable for scenarios where human faces and other images are subject to change. On this basis, the LBP algorithm is improved by adding the center pixel, and the improved LBP algorithm is expressed as CLBP, the LBP operator of the center pixel. CLBP can be written as

(4) $$\begin{array}{c} F_{CLBP}=\overset{p-1}{\underset{p=0}{\sum }}S\left(I_{c},c_{I}\right),S\left(x,c_{I}\right)\text{.} \end{array}$$

In equation (4), F_CLBP_ refers to the CLBP operator, S signifies the symbolic function, *I*_c_ represents the central pixel of the image, and *c*_I_ denotes the average gray value information of the corresponding image.

Due to the rotation and other influencing factors of the image processing, the robustness of CNNs will decrease in the application process. The rotation-invariant characteristics of the LBP algorithm can compensate for the defects of the CNN. Therefore, a facial emotion recognition algorithm is proposed by integrating CNN features with CLBP features. In this hybrid algorithm, feature fusion is completed in the second fully connected layer of the CNN. The specific feature fusion process includes selecting a suitable feature fusion method and the dimensionality reduction operation. Here, the feature fusion method based on connection is adopted, and (5) describes the feature fusion of the two output vectors.

(5) $$\begin{array}{c} consat\left(x,y\right)=\left(x_{1},x_{2},\cdots ,x_{n},y_{1},y_{2},\cdots ,y_{n}\right)\text{.} \end{array}$$

Then, image dimension reduction is realized by principal components analysis to remove the redundant information during image feature fusion. The specific implementation of this step is the centralization of the sample first, as shown in

(6) $$\begin{array}{c} u_{i}=x_{i}-\bar{x}\text{,} \end{array}$$

where $\bar{x}$ represents the average value corresponding to the sample data. The subsequent covariance matrix can be presented as

(7) $$\begin{array}{c} C=\frac{1}{N}\overset{N}{\underset{i=1}{\sum }}{\left(x_{i}-\bar{x}\right)\left(x_{i}-\bar{x}\right)}^{r}=MM^{T}\text{,} \end{array}$$

where *M* represents the matrix corresponding to the sample vector that has been centralized.

Equation (8) indicates the cumulative contribution degree *η* corresponding to the feature value.

(8) $$\begin{array}{c} \eta =\overset{i}{\underset{k=1}{\sum }}\frac{\lambda_{j}}{\overset{h}{\underset{i=1}{\sum }}\lambda_{j}}\text{.} \end{array}$$

In equation (8), *λ*_j_ represents the feature value of the feature matrix, and *h* illustrates the number of feature values. Assume that the feature vector corresponding to the feature value is

(9) $$\begin{array}{c} Z=\left(\eta_{1},\eta_{2},\cdots ,\eta_{t}\right)\text{.} \end{array}$$

Then, the projection of the feature matrix in it can be calculated according to

(10) $$\begin{array}{c} H_{L}=H*Z\text{,} \end{array}$$

where *H*_L_ represents the feature matrix after the dimensionality reduction.

The article "Facial Emotion Recognition Using a Novel Fusion of Convolutional Neural Network and Local Binary Pattern in Crime Investigation" was retracted in 2026. Reasons: suspected computer-generated content; concerns about the data; concerns about the peer review; concerns about the citations.

The neural network fused with the CNN feature and the CLBP feature is represented as hybrid CNN-CLBP model. For the hybrid CNN-CLBP model, the face images of the selected data set are cropped first. Then, the face image samples are rotated and normalized. Besides, the samples are divided into a training set and a test set according to the proportion of 8 : 2. The output facial expression features are input to the Softmax layer to obtain the classification results.  Figure 2 reveals the corresponding structural composition of CNN-CLBP.

### 3.6. Training of the Facial Emotion Recognition Model Based on a Neural Network Algorithm

Static data sets and dynamic data sets are often used to recognize facial expressions, among which JAFFE is a common static image database [32], and CK+ (Cohn-Kanade+) and Fer2013 are image data sets composed of dynamic expression sequences [33, 34]. Considering that facial expression recognition generally processes dynamic expression sequences, the CK+ and JAFFE are chosen as the research data sets.  Table 2 presents the image composition of the two data sets.

In the detection and recognition of facial expressions, the JAFFE data set and the CK + data set are common. In addition, the information contained in these two databases is more comprehensive, which can effectively improve the model performance and the accuracy for facial emotion recognition. Due to facial expressions' dynamic characteristics, images of six typical expressions of the CK + data set are chosen for facial emotion recognition. Some face images of the JAFFE data set are shown in Figure 3. Some face images of the CK + data set are presented in Figure 4.

In addition to selecting data sets, positioning detection is a critical step in recognizing human facial expressions. The accuracy of positioning detection directly impacts the recognition accuracy. Therefore, it is vital to select applicable positioning detection algorithms. In other words, a positioning detection algorithm meeting the requirements needs to consider both accuracy and efficiency. Consequently, the Haar-like algorithm is adopted to describe the facial features of human faces, and the AdaBoost algorithm is adopted for classification. In the process of feature extraction using Haar-like, feature values can be expressed as

(11) $$\begin{array}{c} f_{h}=\left|a\sum_{\left(x,y\right)\in S_{A}}i\left(x,y\right)-b\sum_{\left(x,y\right)\in S_{B}}i\left(x,y\right)\right|\text{,} \end{array}$$

where *S*_*A*_ represents the black composition in the region, and *S*_*B*_ denotes the white composition in the region. Besides, *a* refers to the proportion of the black area in the area, *b* stands for the proportion of the white area in the area, and *i* (*x*, *y*) represents the corresponding pixel value in the image feature interval.

The article "Facial Emotion Recognition Using a Novel Fusion of Convolutional Neural Network and Local Binary Pattern in Crime Investigation" was retracted in 2026. Reasons: suspected computer-generated content; concerns about the data; concerns about the peer review; concerns about the citations.

Furthermore, the feature number can be determined according to

(12) $$\begin{array}{c} SUM=XY\left(W+1-w\frac{X+1}{2}\right)\left(H+1-h\frac{Y+1}{2}\right)\text{.} \end{array}$$

In (12), *W* represents the width of the image, *H* signifies the height of the image, *w* denotes the width of the rectangle, and *h* refers to the height of the rectangle. Meanwhile, *X* represents the magnification factor of the rectangular feature in the horizontal direction, and *Y* stands for the rectangular feature magnification factor in the vertical direction.

For the AdaBoost training strong classifier, *N* training samples are expressed as

(13) $$\begin{array}{c} \left(X_{1},Y_{1}\right),\cdots \left(X_{N},Y_{N}\right)\text{,} \end{array}$$

where *Y*_*i*_ = *0* indicates negative samples of nonface data, and *Y*_*i*_ = *1* refers to positive samples of image data. Then, the weight initialization process is performed. In the case of *Y*_*i*_ = *0*, the weight can be written as (4).

(14) $$\begin{array}{c} W_{i,j}=\frac{1}{2m}\text{.} \end{array}$$

In the case of *Y*_*i*_ = *1*, the weight can be expressed as

(15) $$\begin{array}{c} W_{i,j}=\frac{1}{2l}\text{,} \end{array}$$

where *m* represents the number of negative samples, and *l* denotes the number of positive samples. The normalization of weights can be presented as

(16) $$\begin{array}{c} \frac{W_{i,j}}{\overset{N}{\underset{j=1}{\sum }}W_{i,j}}⟶W_{i,j}\text{.} \end{array}$$

Then, it is necessary to train the model using the features by a weak classifier. The final step of classification using the AdaBoost algorithm is to update the weights. The strong classifier can be expressed as

(17) $$\begin{array}{c} h\left(x\right)=\left\{\begin{array}{cc} 1 & \overset{T}{\underset{t=1}{\sum }}a_{l}h_{l}\left(x\right)\geq \frac{1}{2}\\ 0 & other \end{array}\right.\overset{T}{\underset{t=1}{\sum }}a_{t}\text{,}\\ a_{t}=\log\frac{1}{b_{i}}\text{.} \end{array}$$

Before training the model using images, since the background information on the original image may obstruct recognizing and detecting the image, the image preprocessing mainly contains grayscale processing, cropping processing, and normalization. Generally, the CNN has an excellent performance in image processing, and it is unnecessary to preprocess images or extract features, since the fine-grained feature extraction of CNN can process the images. However, face images usually involve complicated information that is affected by multiple factors, such as the visual angle and background information. Therefore, the image information cannot be exactly exacted by a separate operation. The initial image information is processed via grayscale, cropping, and normalization. The grayscale processing is to convert the color image into a grayscale image with a single channel feature. After this operation, both the influence of light intensity and the calculation complexity in the training process decrease, improving the model's training speed. Specifically, the gray value conversion can be calculated according to

(18) $$\begin{array}{c} 0.299R+0.587G+0.114B=Y\text{,} \end{array}$$

where *R* represents the red channel in the image, *G* denotes the green channel in the image, B refers to the blue channel in the image, and Y stands for the gray value.

The article "Facial Emotion Recognition Using a Novel Fusion of Convolutional Neural Network and Local Binary Pattern in Crime Investigation" was retracted in 2026. Reasons: suspected computer-generated content; concerns about the data; concerns about the peer review; concerns about the citations.

Furthermore, the image cropping is indispensable since there exists a considerable amount of disturbance information on the initial face image, which may reduce classification accuracy. Therefore, the face image is cut before expression recognition. The specific cutting method is that, in the horizontal direction, a crop factor of 0.7 is selected to complete the image cropping process. In the vertical direction, a crop factor of 0.3 is selected to complete the cropping process. After the cropping operation, the information on the image irrelevant to facial expressions is removed, and the size of the image is significantly reduced, which can significantly reduce the workload of the subsequent training. The final part after the cropping processing is the normalization of the image. Specifically, during the normalization processing, the initial image of the data sets is rotated by -30°, -15°, 15°, and 30°, respectively, considering that there may be nonfrontal facial images. Subsequently, facial emotion recognition is performed after the normalization. The image preprocessing mainly aims to reduce the impact of uneven lighting on the facial emotion recognition. In the normalization of the image, the histogram is used to equalize the image, which can be expressed as

(19) $$\begin{array}{c} s_{i}=H\left(n\right)=\overset{k-1}{\underset{i=0}{\sum }}\frac{n_{l}}{n}\text{,} \end{array}$$

where *n* denotes the total number of pixels in the human face image, *k* represents the type of gray value, and *n*_l_ refers to the total amount corresponding to the l-th type of gray value.

The article "Facial Emotion Recognition Using a Novel Fusion of Convolutional Neural Network and Local Binary Pattern in Crime Investigation" was retracted in 2026. Reasons: suspected computer-generated content; concerns about the data; concerns about the peer review; concerns about the citations.

It is essential to use a feasible optimization algorithm to find the model's optimal global solution to train the CNN model. Adam algorithm is an optimization algorithm developed based on a stochastic gradient algorithm. The algorithm has the characteristics of an adaptive gradient and root mean square propagation. The adaptive gradient provides the algorithm with excellent performance in computer vision, and root mean square propagation affords the algorithm excellent performance in solving intermittent problems. The mean value of the initial time gradient in the Adam algorithm can be obtained according to

(20) $$\begin{array}{c} \hat{M_{t}}=\frac{M_{l}}{1-b_{1}^{l}}\text{.} \end{array}$$

The noncentral variance corresponding to the gradient at the second moment can be expressed as

(21) $$\begin{array}{c} \hat{V_{t}}=\frac{V_{l}}{1-b_{2}^{l}}\text{,} \end{array}$$

where $\hat{M_{t}}$ indicates the mean value of the corresponding gradient at the initial time, *b*_1_ = 0.9, $\hat{V_{t}}$ represents the noncentral variance of the corresponding gradient at the second time, and *b*_2_ = 0.999.

This algorithm updates the parameters according to

(22) $$\begin{array}{c} \theta_{t+1}=\theta_{I}=\frac{\eta }{\sqrt{\hat{V_{t}}+\varepsilon }}\hat{M_{t}}\text{.} \end{array}$$

The Adam algorithm has excellent convergence performance and requires a small amount of memory space. Therefore, the algorithm can solve optimization problems, including numerous data information and parameters [35]. Therefore, the algorithm is selected as a tool to optimize the neural network.

The cross-entropy loss function can measure and evaluate the difference between the probability distributions. Here, this function presented in (23) is selected as the loss function.

(23) $$\begin{array}{c} h\left(p,q\right)=-\underset{x}{\sum }p\left(x\right)\log\;q\left(x\right)\text{.} \end{array}$$

In equation (24), *p* refers to the correct probability distribution value, and *q* represents the predicted value. Furthermore, discrete variables can be calculated according to

(24) $$\begin{array}{c} h\left(p,q\right)=\underset{x}{\sum }p\left(x\right)\cdot \log\left(\frac{1}{q\left(x\right)}\right)\text{.} \end{array}$$

Continuous variables can be decided according to

(25) $$\begin{array}{c} -\int_{x}p\left(x\right)logq\left(x\right)dr\left(x\right)=E_{p}\left[-\log\;q\right]\text{.} \end{array}$$

The article "Facial Emotion Recognition Using a Novel Fusion of Convolutional Neural Network and Local Binary Pattern in Crime Investigation" was retracted in 2026. Reasons: suspected computer-generated content; concerns about the data; concerns about the peer review; concerns about the citations.

### 3.7. Comparative Experiment

The CK + data set is chosen to verify the effectiveness of the hybrid CNN-CLBP model. On the premise of ensuring that all training parameters are consistent, the average and maximum values are used as comparison indicators. The hybrid CNN-CLBP model is compared with the traditional machine learning LBP model, a single LeNet-5 model, and a single VGGNet model.  Table 3 provides the particular parameter settings of the LeNet-5 model and the VGGNet model.

For the facial emotion recognition algorithm based on feature fusion, after a series of preprocessing operations on the image, quantitative analysis is performed on the three indicators of accuracy, cross-entropy, and loss function to test the effectiveness of the feature fusion method.

## 4. Results

### 4.1. Comparative Analysis of Facial Emotion Recognition Results

Figure 5 indicates the facial emotion recognition results of the hybrid CNN-CLBP model, the traditional machine learning model LBP, the LeNet-5 model, and the VGGNet model.

From Figure 5(a), the average recognition rate of the traditional machine learning LBP model reaches 48.63%, that of the single LeNet-5 model is 73.22%, that of the single VGGNet network model attains 83.17%, and that of the hybrid CNN-CLPB model attains 88.16%. By the traditional machine learning model LBP, the recognition rates of the three emotions of anger, sadness, and fear are 32.31%, 28.71%, and 24.08%, respectively. In contrast, the single LeNet-5 model achieves a higher recognition rate for each expression than the traditional machine learning LBP model. On the whole, the hybrid CNN-CLPB model has a significant advantage in the recognition rate. Therefore, the hybrid CNN-CLPB model has the best effect on facial emotion recognition among the comparative models.

Figure 5(b) displays the comparison of the mean values and maximum values of facial emotion recognition for each expression by the hybrid CNN-CLPB model, the traditional machine learning LBP model, the LeNet-5 model, and the VGGNet model.

In Figure 5(b), the traditional machine learning LBP model has the highest recognition rate for the facial emotion of surprise, reaching 73.2%, and the LeNet-5 model has the highest recognition rate for happiness, reaching 86.77%. Moreover, the VGGNet model has the highest recognition rate for happiness of 94.11%. Ultimately, the hybrid CNN-CLPB model also has the highest recognition rate for happiness, reaching 98.61%.

### 4.2. Quantitative Analysis of the CNN-CLBP Model Based on Feature Fusion

The accuracy, cross-entropy, and loss function of the hybrid CNN-CLBP model on the training set and the test set are shown in Figure 6.

The article "Facial Emotion Recognition Using a Novel Fusion of Convolutional Neural Network and Local Binary Pattern in Crime Investigation" was retracted in 2026. Reasons: suspected computer-generated content; concerns about the data; concerns about the peer review; concerns about the citations.

According to the analysis of the data changes in Figure 6, the accuracy rate trend of the CNN-CLBP model on the training set is almost identical to that on the test set, and the entire training process is stable. When the corresponding training steps are less than 2k, the accuracy rate of the model on the test set shows an exponential changing trend. When the corresponding training steps are within the range of 4k–8k, the accuracy rate of the model on the test set still shows relatively rapid growth. When the training steps fluctuate around 8k, the accuracy rate of the model on the test set reaches 96.8%, and then, it tends to be stable. At this time, the recognition rate of facial emotions is extremely high. There is no obvious deviation from the changing trend of cross-entropy of the training set to that of the test set. The prediction distribution of the model on the test set is closer to the actual value. When the training steps are around 8k, the corresponding value of the cross-entropy shows a small reduction. Then, the corresponding value of cross-entropy is continuously decreasing as the training step increases. For the changes in the loss function, when the training step increases, the function value of the model on the test set continues to decrease. When the number of iterations reaches 20k, the value of the function gradually stabilizes. In this quantitative analysis, both the training set and the test are set to cover all participants in the data set, but the images are chosen randomly.

### 4.3. Facial Emotion Recognition Analysis of the CNN-CLBP Model

Based on the CK + data set, the hybrid CNN-CLBP model recognizes typical facial expressions on face images, including anger, disgust, fear, happiness, sadness, and surprise. The results are shown in Figure 7. The facial emotion recognition effects of the hybrid CNN-CLBP model are presented in Figure 8.

Through Figure 7, the hybrid CNN-CLBP model provides a higher recognition rate of the expression of happiness and surprise than of the other expressions. Moreover, the average recognition rate of the facial expression of sadness is the lowest, reaching 77.46%. The probability of erroneous judgment as sadness is 9.50%, and the probability of erroneous judgment as disgust is 6.18%.

## 5. Discussion

Different from psychologically and physiologically mature adults, juveniles are in a critical developing period of physical and mental maturity. Hence, it is vital and essential to pay attention to juveniles, especially the psychology of juveniles involved in crime. Emotion recognition is a critical method based on psychoanalysis. In summary, the recognition rate of facial expressions by the traditional machine learning LBP model is significantly different from the current recognition algorithms for facial expressions. The reason is that the operator of the traditional machine learning LBP model is a matching algorithm focusing on analyzing the differences between different categories, thereby leading to the loss of detailed information on the image.

The article "Facial Emotion Recognition Using a Novel Fusion of Convolutional Neural Network and Local Binary Pattern in Crime Investigation" was retracted in 2026. Reasons: suspected computer-generated content; concerns about the data; concerns about the peer review; concerns about the citations.

However, facial expressions are precise reflections of the details. The image contains complex and nuance information, so the traditional machine learning LBP model has a low effect on recognizing facial expressions. The hybrid CNN-CLBP model significantly ameliorates the recognition accuracy of facial expressions. The reason is that more convolutional layers in the model can greatly improve its ability to indicate image features and reflect the detailed information on the image more accurately.

There are many research results of the application of deep learning to facial expression recognition, including the application of CNN and LBP, as shown in Table 4.

In facial emotion recognition, the hybrid CNN-CLBP model effectively avoids the problem that traditional models are easily affected by the number of network layers. Facial emotion recognition is affected by many problems caused by image rotation. The effective fusion of CNN features and CLBP features deals with such problems easily. In addition to the VGGNet model, the recognition accuracy of hybrid CNN-CLBP model is significantly better than other classical models, which may be related to the number and structure of the convolutional layers in the network. As a result, the hybrid CNN-CLBP model has achieved marvelous applicability to recognizing facial expressions, providing satisfying results of the classification of facial emotions and expressions. Meanwhile, the psychological changes of juveniles involved in crimes are also a manifestation of emotional changes closely related to their facial expressions. The hybrid multilayer CNN-CLBP model shows excellent performance in recognition of facial emotions. It provides an important development direction for analyzing psychological changes and the extraction of psychological characteristics of juveniles involved in crimes. In the recognition process of facial expressions and emotions, the training set and the test set of the hybrid CNN-CLBP model show a similar changing trend, and there is no significant difference between the changing trends of test accuracy rate and the training accuracy rate. In other words, poor-fitting never occurs, which shows that the preprocessing of face images is sufficient, and the optimization of neural network model parameters further ensures the stability of the training process. In contrast, LBP is improved by this work to expand the application of deep learning method for facial expression recognition.

The article "Facial Emotion Recognition Using a Novel Fusion of Convolutional Neural Network and Local Binary Pattern in Crime Investigation" was retracted in 2026. Reasons: suspected computer-generated content; concerns about the data; concerns about the peer review; concerns about the citations.

In summary, it is obvious that the combination of LBP and CNN has achieved some research results in facial expression recognition, but the fusion of CNN and CLBP in facial expression recognition is still relatively scarce, which is an innovative trait of this paper. Furthermore, the hybrid CNN-CLBP model is applied here to identify facial expressions, which further expands the application field of the deep hybrid model. The effectiveness of the overall emotion recognition can be confirmed through the preprocessing and recognition of the images.

From the perspective of facial expression recognition, the hybrid CNN-CLBP model has a high recognition accuracy for the two expressions of happiness and surprise, and the probability of erroneous judgment as the expression of sadness is large. This indicates that the emotional expression of sadness in the pixel space cannot be effectively separated from other expressions. The reason may be that changes in expressions such as happiness and surprise have more significant characteristics. The amplitude of such expression changes is more extensive, which is easier to distinguish and identify. Besides, the emotional performance of happiness and surprise is different from other types of emotions. Since the connection between them is not apparent, the model shows higher recognition rates for these two emotions. In addition to the weaker changes, the expression of sadness is more likely to come up with expressions of negative emotions such as disgust and fear. Under the premise of such an obvious correlation and high similarity, it is possible to obtain a wrong recognition result. Nevertheless, for the particular group of juveniles, the change in their psychological characteristics is closely related to facial expressions. Thus, understanding their emotions through facial expressions is crucial to exploring their psychological characteristics.

Intelligent learning methods like deep learning have great potential to explore the increasingly severe psychological problems that people are experiencing at all stages. Jiang et al. analyzed the body mass index (BMI) and realized the visual estimation of BMI based on machine learning and computer vision, thus revealing the applicability of deep learning in BMI estimation [44]. Ashiquzzaman et al. proposed an optimized deep learning convolutional neural network (DCNN). By introducing the spatial pyramid layer, the authors maintained the input dimension of DCNN at a fixed level, with faster computing speed and good performance in gesture detection and recognition. The above works laid the foundation for the application of human-computer interaction based on gesture input [44]. The potential psychological conditions or psychological problems are tapped from the perspective of facial emotion recognition here [45–48]. This method is not perfectly accurate, but emotion is an externalized expression of people's psychological states, so analyzing the psychological states through emotion is a feasible way [49–52]. This is also consistent with the above research results [53]. Besides, paying attention to juveniles' psychological states, especially those involved in crimes, and giving appropriate psychological guidance and method guidance have a positive role in helping juveniles establish correct outlooks on life and values [54–57]. The hybrid CNN-CLBP model reported here achieves excellent performance in facial expression recognition and can precisely capture different facial expressions. This is beneficial to judging changes in the psychological states of juveniles via facial expression recognition. In addition, the combination of emotion recognition through facial expressions with psychological analysis also provides a possible direction for extracting and analyzing psychological features.

The article "Facial Emotion Recognition Using a Novel Fusion of Convolutional Neural Network and Local Binary Pattern in Crime Investigation" was retracted in 2026. Reasons: suspected computer-generated content; concerns about the data; concerns about the peer review; concerns about the citations.

## 6. Conclusions

By applying the hybrid CNN-CLBP model to facial emotion recognition, the essential conclusions are drawn as follows. Increasing the number of network layers of CNN can effectively improve expression recognition accuracy. Besides, image preprocessing and parameter optimization have a significant effect on enhancing the effectiveness of the model. Moreover, the hybrid CNN-CLBP model shows quite exceptional results in the fusion of facial image features and has the best accuracy in recognizing the facial expressions of happiness and surprise. The emotion recognition depending on facial expression and guided by the connection between emotion and psychology provides a direction for the simple analysis of psychological characteristics of juvenile criminals and initially combining deep learning methods with psychoanalysis.

However, several shortcomings have been identified. The hybrid CNN-CLBP model can extract relevant feature data onto expressions, but it cannot investigate particular psychological characteristics. Therefore, in the future, psychological counseling and other elements will be included to analyze and explore the psychological characteristics of juvenile criminals in a profound and detailed manner.

## Figures and Tables

**Figure 1:** Structure of CNN.

**Figure 2:** Structure of the hybrid CNN-CLBP model.

**Figure 3:** Human face images of the JAFFE data set (the data source: https://blog.csdn.net/akadiao/article/details/79956952).

The article "Facial Emotion Recognition Using a Novel Fusion of Convolutional Neural Network and Local Binary Pattern in Crime Investigation" was retracted in 2026. Reasons: suspected computer-generated content; concerns about the data; concerns about the peer review; concerns about the citations.

**Figure 4:** Human face images of the CK + data set (the data source: https://blog.csdn.net/yinghua2016/article/details/77323537).

**Figure 5:** Comparison of recognition results of several facial emotion recognition methods: (a) recognition rate; (b) recognition results and time consumption.

**Figure 6:** Quantitative analysis results of the CNN-CLBP model based on feature fusion.

**Figure 7:** Facial emotion recognition results of the hybrid CNN-CLBP model.

**Figure 8:** Facial emotion recognition effects of the hybrid CNN-CLBP model (the picture material comes from the public face recognition data set on the web page).

**Table 1:** Parameter settings of the facial emotion recognition neural network based on psychological feature analysis.

Network structure	Convolution layer	Pooling layer	Fully connected layer	Output layer
Output size	1 : 128∗128∗1	1 : 28∗28∗6	1 : 1∗1∗1	1∗1∗6
	2 : 64∗64∗1	2 : 10∗10∗16	2 : 1∗1∗6	
	3 : 32∗32∗1			
	4 : 14∗14∗6			

**Table 2:** Image composition of Fer2013 and CK + data sets.

Datasets	JAFFE	CK+
Image composition	Number of images: 35886	Number of images: 593
	Size: 48∗48 pixel	Size: 640∗480 pixel
	Participants: 10	Participants: 123
	Tags: happy, fear, sad, surprised, angry, disgusted, neutral	Tags: happy, fear, sad, surprised, contempt, anger, disgust, neutral

**Table 3:** Parameter settings of LeNet-5 and VGGNet models.

Network layer		Input size	Convolution kernel size	Output size
Lenet-5	Convolution layer 1	32∗32∗1	5∗5∗1	28∗28∗4
	Lower sampling layer 1	28∗28∗4	2∗2	14∗14∗4
	Convolution layer 2	14∗14∗4	5∗5∗6	10∗10∗14
	Lower sampling layer 2	10∗10∗14	2∗2	5∗5∗14
	Convolution layer 3	5∗5∗14	5∗5∗14	1∗1∗120
	Full connection layer	1∗1∗120	120∗82	1∗1∗82
	Output layer	1∗1∗82	82∗10	1∗1∗10
VGGNet	Convolution layer 1	224∗224∗3	11∗11∗3	55∗55∗46
	Lower sampling layer 1	55∗55∗46	3∗3	27∗27∗46
	Convolution layer 2	27∗27∗46	5∗5∗46	27∗27∗128
	Lower sampling layer 2	27∗27∗126	3∗3	13∗13∗128
	Convolution layer 3	13∗13∗126	3∗3∗256	13∗13∗192
	Convolution layer 4	13∗13∗192	3∗3∗192	13∗13∗192
	Convolution layer 5	13∗13∗192	3∗3∗192	13∗13∗128

**Table 4:** Comparison of research based on algorithm recognition.

Author	Primary research contents
Jain et al. [36]	They constructed a facial expression recognition system based on a single deep CNN, including a convolution layer and a deep residual layer. Through the training of face image labels and the training of CK + dataset and JAFFE dataset, they found that the model with deep convolution layer had better recognition effect and accuracy than the traditional emotion recognition methods.
Ma and Celik [37]	They proposed a densely connected CNN structure applicable to facial expression recognition, and through this structure, the output and input of adjacent convolution layers were connected. They finally verified the effectiveness of the structure in facial expression recognition.

*These works provide solid support for the research work reported here and reveal the effectiveness and necessity of this research work.*	
Liu et al. [38]	They applied the fused CNN and CLBP to intelligent mining. By considering the unique visual features, they found that, in the case of applying the fused model, the accuracy of image recognition could be improved by 2% to 3% compared with the traditional methods.
Shao and Qian [34]	They proposed a two-branch CNN model. By extracting traditional LBP features and deep learning features, they found that the fusion of LBP features and CNN showed excellent performance and applicability in facial expression recognition.
Takalkar et al. [39]	They combined LBP with CNN for microexpression recognition. Through the evaluation of seven widely used microexpression databases, they found that the recognition accuracy of the proposed method had been significantly improved, and the relevant training and testing could be realized through a small number of data sets.

*In contrast, this work further optimizes LBP and extends the application of deep learning method to facial expression recognition.*	
Liu and Zhang [40]	They found that the recognition accuracy of CNN model could reach 78.9% after analyzing the accuracy of deep neural network in image recognition on CK + data set.
Shahid et al. [41]	They proposed a multiclass SVM and topic-related k-fold crossover method for facial expression recognition. They found that the recognition rate of this method for CK + data set could reach more than 90%, and the accuracy and calculation time were improved.
Liao et al. [42]	They introduced the conditional random forest structure to build a deep multi-instance learning model. They found that, in the field of automatic facial expression recognition, the recognition rate of the model on CK + public data set could reach more than 86%.
Miyoshi et al. [43]	They proposed an enhanced convolutional long short-term memory algorithm for automatic facial expression recognition. The test results showed that the recognition accuracy of this algorithm on CK + data set was more than 85%.
Hybrid CNN-CLBP algorithm reported here	In conclusion, although the recognition rate of the hybrid CNN-CLBP algorithm is lower than that proposed in [41], the average recognition rate for different types of expressions is still more than 88%, which is better than the current advanced algorithms. At the same time, this algorithm also considers the relationship between expression recognition and psychological analysis, which is different from other studies.

The article "Facial Emotion Recognition Using a Novel Fusion of Convolutional Neural Network and Local Binary Pattern in Crime Investigation" was retracted in 2026. Reasons: suspected computer-generated content; concerns about the data; concerns about the peer review; concerns about the citations.

## Data Availability

The raw data supporting the conclusions of this article will be made available by the authors, without undue reservation.
